The article "Water droplet on inclined dusty hydrophobic surface: influence of droplet volume on environmental dust particles removal" was retracted in 2026. Reasons: unreliable results or conclusions; concerns about the data.

# Water droplet on inclined dusty hydrophobic surface: influence of droplet volume on environmental dust particles removal

**DOI:** 10.1039/c8ra10092f

**Published:** 2019-01-28

**Authors:** Ghassan Abdelmagid, Bekir Sami Yilbas, Abdullah Al-Sharafi, H. Al-Qahtani, Nasser Al-Aqeeli

**Affiliations:** Mechanical Engineering Department, King Fahd University of Petroleum & Minerals Dhahran Saudi Arabia bsyilbas@kfupm.edu.sa; Center of Excellence in Renewable Energy, King Fahd University of Petroleum & Minerals Dhahran Saudi Arabia

## Abstract

A water droplet's behavior on an inclined hydrophobic surface in the presence of environmental dust particles is considered and the droplet's dynamics are analyzed pertinent to self-cleaning applications. A polycarbonate wafer is crystallized using the solution-crystallization method to generate hierarchically distributed micro/nano-sized spherules and pillars on the surface. To improve the wetting state and lower the contact angle hysteresis, functionalized silica particles are synthesized and, later, deposited on the crystallized surface. Environmental dust particles are collected and characterized in terms of elemental composition, size and shape. A high-speed camera is used to monitor a water droplet's behavior on the inclined hydrophobic surface with and without the presence of dust particles. The influence of droplet volume on the dust particle removal rate from the inclined hydrophobic surface is assessed. It is found that the functionalized silica particles deposited on the surface result in a droplet contact angle in the order of 158 ± 2° and contact angle hysteresis of 2 ± 1°. The water droplet mainly rolls on the inclined hydrophobic surface and the sliding velocity remains almost 13% of the transverse velocity of the droplet. Droplet wobbling is influenced by the dust particles and the droplet size; in which case, increasing the droplet volume enhances the droplet puddle thickness on the hydrophobic surface. The cloaking of the droplet fluid onto the dust particles causes mixing of the dust particles with the droplet fluid while enhancing the particle removal from the hydrophobic surface. Increasing the droplet volume slightly enhances the size of the area of the cleaned surface.

## Abstract 2

A water droplet's behavior on an inclined hydrophobic surface in the presence of environmental dust particles is considered and the droplet's dynamics are analyzed pertinent to self-cleaning applications.

## Introduction

The hydrophobic wetting state remains a demanding surface characteristic in self-cleaning applications. This is because pinning forces associated with the adhesion of the particles on the hydrophobic surface remain small. In general, hydrophobic surfaces have a hierarchically distributed textured topology consisting of micro/nano pillars with low free energies. The air trapped in between the textured pillars reduces the contact area between the particles and the surface; in addition, interatomic and molecular attraction forces between the particles and the surface decrease as the surface free energy reduces. Consequently, a combination of reduced contact area, due to air gaps, and low atomic and molecular interaction forces between the particles and the surface enables a reduction in the efforts required to remove the particles from the surface. One of the challenges of creating hydrophobic surfaces is fulfilling the requirements of the hierarchically distributed textured topology. Several methods have been introduced towards achieving a surface textured topology with a hydrophobic wetting state. In general, the strategies mimic nature by creating a surface texture similar to those of lotus leaves, rose petals, rice leaves, or similar. In some cases, surface texturing involves multi-step processes and requires expensive or hazardous specialized agents. Some of the types of surface processing towards achieving a hydrophobic wetting state include: phase separation,^1^ electrochemical deposition,^2^ plasma treatment,^3^ sol–gel processing,^4^ electrospinning,^5^ laser texturing,^6^ and solution immersion.^7^ However, a simple and one-step surface process for achieving the hydrophobic state is demanded. The fabrication of hydrophobic surfaces towards creating self-cleaning effects on surfaces was one focus of interest.^8–20^ A hydrophobic organic layer on a surface could be formed *via* chemical etching, followed by the deposition of oxide nanoparticles.^8^ The resulting wetting state of the coating surface could be further increased by depositing a thin layer of organic molecules on the coating surface.^9^ The introduction of chemical etching and stearic acid modification on aluminium surfaces resulted in a hydrophobic state of the surface, which was favourable in terms of environmentally friendly green processing and a short processing time.^10^ The robustness of the surface texturing for self-cleaning applications played a critical role in selecting the appropriate processes; in which case, an amphiphobic coating which created flower-like nanostructures on the micro-patterned polymer substrate became favourable for its low hysteresis and high contact angle of the droplets.^11^ However, the process could involve long duration and high cost. One of the challenges in the wetting state of the surface was keeping the surface optically transparent, which was particularly important for energy harvesting devices such as photovoltaic and solar thermal power systems. Introducing an optically corrected fluid, such as silicon oil, by impregnation on the textured surface could improve the optical transmittance.^12^ Self-cleaning surfaces also found applications in membrane technology.^13^ A novel self-cleaning membrane in the water desalination process was demanded; in which case, self-cleanable membranes composed of nanocellulose and TiO_2_ nanoparticles became favourable.^14^ However, the durability of the hydrophobic coating for self-cleaning applications remained challenging. The hydrophobic coating produced from a mixture of nano-sized TiO_2_, attapulgite (epoxy resin), and polydimethylsiloxane was found to be durable, retaining its self-cleaning ability under wearing environments.^15^ On the other hand, the hydrothermal process could be used in the fabrication of hierarchical CuO spheres on polyimide substrates, which was reported to involve a simple process and could be used effectively for the self-cleaning of organic and inorganic particulates from surfaces.^16^ Sol–gel processing also created a hydrophobic wetting state at the surface, which could be used for self-cleaning applications;^17^ however, the durability of the resulting sol–gel coating in self-cleaning applications was not promising. A copper-based coating could produce superhydrophobic surfaces with long-term durability for self-cleaning applications.^18^ Model studies of hydrophobic surfaces in relation to textural parameters remained important when designing surfaces for self-cleaning purposes.^18,20^ The different length scales of the surface texture resulted in different droplet contact angles and hysteresis, which was demonstrated to be critical to the hydrophobic characteristics of surfaces.^19^ A model study also predicted that the three-phase contact length varied while causing the droplet to spread as the droplet volume changed.^20^

On the other hand, environmental dust storms had detrimental effects on surfaces: in particular, surfaces with optical and sensitive air friction characteristics, such as selective surfaces for energy harvesting devices and aircraft bodies. Although the elemental composition of the environmental dust particles depends on the local geological structures of the geographic landscape, alkaline and alkaline earth metals remained common in the dust particles. In humid ambient conditions, water condensed onto the dust particles and formed a chemically active liquid solution *via* dissolution of the alkaline and alkaline earth metals of the dust compounds in the water condensate. The liquid solution impregnated the solid surface under gravitational influence. A film was formed by the liquid solution and it had multi-fold effects on the surfaces; in which case, chemical activities caused the initiation of erosion and corrosion sites on the surface. In addition, upon drying, the liquid solution formed an interlayer between the dust particles and the surface. The efforts required to remove the dust particles from such surfaces became significantly high.^21^ Dust particle mitigation around the globe has been investigated previously;^22^ however, the prevention of the after-effects of dust storms is still under investigation. Dust particle adhesion on surfaces was an important factor for self-cleaning applications.^23^ It was demonstrated that the mud formed from a mixture of water condensate and the dissolved dust particles had prime importance for self-cleaning applications of surfaces, which became significant in humid ambient conditions.^24^ In the case of metallic materials, dust accumulation on surfaces and its after-effects became critical to maintaining the surface integrity in terms of roughness and texture size because of erosion and corrosion sites developing on the surface.^25^ However, the hydrophobic texturing of metallic surfaces suppressed the erosion and corrosion on the surface by lowering the dust particle adhesion.^26^ In addition, a chemically passive layer developed during surface texturing, such as the formation of nitride species, suppressed the corrosion and erosion influence of the dust solution on the surfaces.^27^

Although dust particle removal from hydrophobic surfaces towards self-cleaning applications was studied previously,^28^ the main focus was to investigate the droplet dynamics on a hydrophobic surface and water droplet cloaking of the dust particles for a constant water droplet volume. The influence of the droplet volume on the dust removal mechanisms from inclined hydrophobic surfaces was left for future study. In addition, the droplet wobbling and the droplet puddle thickness on a hydrophobic surface change with the droplet volume during rolling, which in turn alters the size of the three-phase-contact line and the contact angle hysteresis on the surface. This behaviour influences the droplet dynamics on the surface and the amount of dust particles removed, by the rolling droplet, changes. Consequently, the effectiveness of the self-cleaning process changes with the droplet volume on the inclined hydrophobic surface. In the present study, the influence of water droplet size on dust particle removal from a hydrophobic surface is considered and the water droplet dynamics on the inclined hydrophobic surface are investigated in relation to self-cleaning applications. The properties of dust particles collected from the local environment are examined in terms of elemental composition, density, size and shape. The droplet rolling and sliding mechanisms on the hydrophobic surface are analysed by including different sizes of droplets. The effectiveness of droplet dust removal from the surface is introduced to assess the efficacy of the cleaning of the hydrophobic surface by the water droplet.

## Experimental

The experimental procedures and characterization tools used in the experiments are provided under the following relevant headings.

### Solution crystallization of polycarbonate surface and functionalized silica particle deposition

Polycarbonate samples with dimensions of 30 mm × 250 mm × 3 mm (width × length × thickness) were prepared for the surface crystallization. The samples were cleaned ultrasonically before immersion into an acetone bath. However, several tests were conducted to select the right combination of acetone concentration and immersion time to achieve hierarchically distributed micro/nano spherules and fibrils on the sample surface through the solution-crystallization process, in line with the earlier study.^29^ Consequently, optimum process parameters were identified and used in the crystallization of the sample surfaces. These parameters included acetone volumetric concentration (60%) and immersion time (3 minutes). The wetting state of the solution-crystallized surface resulted in a droplet contact angle in the order of 130° ± 4° with contact angle hysteresis of 36° ± 2°. In order to improve the wetting state of the surface in terms of increasing the contact angle and reducing the contact angle hysteresis, nano-sized functionalized silica particles were deposited onto the crystallized surface. The nano-sized silica particles were synthesized by using a similar procedure to that reported in the previous study.^30^ During the synthesis and functionalizing cycle for the nano-sized silica particles, tetraethyl orthosilicate (TEOS), isobutyltrimethoxysilane (OTES), ethanol, and ammonium hydroxide were used. The solvent casting method was applied to deposit the functionalized silica particles on the crystallized polycarbonate surface. Vacuum drying was used to remove all of the solvent residues from the surface. The dynamic contact angle of the resulting surface was measured in line with a previous study,^31^ and a contact angle in the order of 158° ± 2° with contact angle hysteresis in the order of 2° ± 1° were measured. This arrangement provided droplet rolling/sliding on the resulting hydrophobic surface. Consequently, the deposition of the functionalized silica particles on the crystallized polycarbonate surface resulted in a hydrophobic surface with a significantly high contact angle and reduced contact angle hysteresis.

### Characterization equipment

SEM (JEOL 6460) and energy dispersive spectroscopy (EDS) were used to examine surface morphology and elemental composition. X-ray photoelectron spectrometry (XPS) was performed using an ESCALAB 220 XL spectrometer. A monochromatic Al K_α_ X-ray source (1486.6 eV) was operated in the constant analyzer energy mode (CAE = 100 eV for survey spectra and CAE = 40 eV for high resolution spectra). X-ray diffraction (XRD, Model: D8 Advanced diffractometer, Manufacturer: Bruker, USA) analysis was performed with CuKα radiation at typical settings of 40 kV and 30 mA. The water droplet motion on the inclined hydrophobic surface and water cloaking of the dust particles were monitored using a high-speed camera (Model: SpeedSense 9040, Manufacturer: Dantec Dynamic, Denmark). Atomic force microscopy/scanning probe microscopy (AFM/SPM) in contact mode were used to analyze the surface texture. The tip was made of silicon nitride with the tip radius in the range of *r* = 20–60 nm. A linear micro-tribometer (MCTX-S/N: 01-04300) was used to measure the tangential force required to remove the functionalized silica particles from the solution-crystallized polycarbonate surface. During the tests, the equipment was set at a contact load of 0.03 N and an end load of 5 N. The scanning speed was 5 mm min^−1^, and the loading rate was 1 N s^−1^. The water droplet contact angle of the solution-crystallized and nano-sized silica particle deposited surfaces were measured using a goniometer in line with the previous study.^31^ During the measurements, the droplet volume was controlled by an automatic dispensing system with a volume step resolution of 0.1 μl. The droplet contact angle measurements were repeated five times at different locations on the surface, ensuring the repeatability of the measurements and uniformity of the surface wetting state.

### Environmental dust particle collection and assessments

The dust particles were collected over a period of 12 months from the local region of Dammam in Saudi Arabia. The particles were collected from photovoltaic panel surfaces through removal by soft brushes and the collected particles were stored in an airtight container. The dust particles collected were later examined in terms of density, size, shape, and elemental composition. It should be noted that the dust particles collected over the 12 month period had similar characteristics in terms of elemental composition, size distribution, and shape.

## Results and discussion

The droplet rolling and sliding on the inclined hydrophobic surface are examined in relation to self-cleaning applications. The influence of the droplet volume on dust particle removal from the hydrophobic surface is presented. The predictions of droplet movement using analytical formulations are compared with those obtained from the experiments.

### Characteristics of crystallized and functionalized silica particle deposited surface

Fig. 1 shows the crystallized polycarbonate surface prior to silica particle deposition. The crystallized surface demonstrates spherules and fibrils, which are protruding from the surface. The spherules are hierarchically distributed on the surface. The nano-sized fibrils emanate from the spherule surface because of acetone diffusion into the surface from the nano-sized pores.^32^ The presence of fibrils alters the surface texture characteristics of the spherules; in which case, small-sized textures are observed on the spherule surfaces. This enhances the lotus effect on the crystallized surface.

**Fig. 1:** SEM micrograph of solution-crystallized polycarbonate surface. The large circle represents spherules and the small circle shows fibrils on the crystallized surface.

Fig. 2 shows an AFM micro-image of the crystallized surface (Fig. 2a) together with a surface line scan (Fig. 2b). The line scan demonstrates the spherule heights, which extend up to 6.5 μm; in this case, secondary crystallization on the surface is responsible for the formation of large-sized spherules on the surface.^32^ In addition, the presence of fibrils is also evident from the AFM line scan (Fig. 2b), appearing as small-amplitude oscillations on the spherule hills. The average roughness of the crystallized surface is in the order of 4.2 μm. In the case of the silica particle deposited surface, Fig. 3 depicts the SEM image of the surface. The surface morphology consists of closely spaced nano-sized particles, which form a textured structure on the surface. The surface roughness is in the order of 160 nm. However, in order to assess the texture characteristics on the surface, silica particles are deposited onto the plain glass surface and the surface characteristics are assessed by the line scan of the AFM probe. This can be seen from Fig. 4, in which the micro-image (Fig. 4a) and line scan (Fig. 4b) obtained from the atomic force microscopy image are shown for the silica particles deposited on the glass surface. Some void-like structures are observed at the surface among the agglomerated nano-sized particles. However, the void-like structures are unevenly distributed over the surface and they are not connected with the porous-like channels or passages.

**Fig. 2:** Atomic force microscopy (AFM) image and line scan across the solution-crystallized polycarbonate surface: (a) two-dimensional image of the crystallized surface, and (b) line scan along the crystallized surface.

**Fig. 3:** SEM micrograph of functionalized silica particle deposited crystallized polycarbonate surface. Pore-like structures are marked with red circles.

**Fig. 4:** Atomic force microscopy (AFM) image and line scan across the functionalized silica particle deposited glass surface: (a) two-dimensional image of the functionalized silica particle deposited surface, and (b) line scan along the functionalized silica particle deposited surface.

The agglomeration of the nano-sized particles is related to the modifier silane, which results in side reactions during functionalization, and the condensation of silane on the silica particle surface triggers the agglomeration of silica particles.^33^ The air gap filling the void-like structure influences the surface hydrophobicity. The adhesion of the silica particles on the glass surface is verified through scratch tests. Fig. 5a shows the tangential force required for the removal of the silica particle coating from the glass surface. It is evident that the silica particles attach strongly to the surface. This can also be seen from the micro-image of the scratch marks (Fig. 5b); in which case, the scratch tester indentation partially removes the silica particles from the surface but some small silica particles remain attached on the glass surface during surface scratching. On the other hand, the wetting state of the surface is assessed using the contact angle measurements with the goniometer; in which case, the measurements are carried out in line with the previous study.^31^

**Fig. 5:** Tangential force measured by a micro-tribometer for silica particle removal from the glass surface and an optical image of the scratch mark: (a) tangential force, and (b) optical image of the scratch mark. Residues of functionalized silica particles on the indentation path.

The crystallized surface results in a water droplet contact angle of about 130° ± 4° and contact angle hysteresis in the order of 36° ± 2°. It is evident that the contact angle hysteresis remains high and the droplet rolling and sliding are suppressed by the large hysteresis angle on the surface. However, the functionalized silica particle deposited surface reveals that the water droplet contact is in the order of 158° ± 2° and the contact hysteresis is about 2° ± 1°. Hence, deposition of the silica particles on the crystallized polycarbonate surface not only increases the droplet contact angle, but lowers the contact angle hysteresis, which is critical for the droplet rolling and sliding on the surface. The contact angle measurements are repeated for several locations on the surface and the variation in the contact angle remains less than 2%. Consequently, the functionalized silica particle deposited surface demonstrates an almost uniform wetting state across the surface.

### Dust particle characteristics

The dust particles are collected from the local area of Dammam in the Kingdom of Saudi Arabia. Fig. 6 shows the SEM micrograph of the dust particles. The dust particles possess different shapes and sizes (Fig. 6a). The average size of the dust particles is measured and is found to be 1.2 μm. The small dust particles attach at the surface of the large-sized dust particles and form clusters (Fig. 6b). The attachment of the small dust particles is related to the particle charges, which develop during the long duration of their stay in air. In this case, small particles are exposed to a long duration of solar irradiation and may form charged compounds, such as non-stoichiometric alkaline and alkaline earth metal compounds of chlorine in an environment near the sea.^34^ The shape of the dust particles may be classified through the shape factor and the aspect ratio.^35^ The shape factor is attributed to the ratio of the dust particle perimeter squared over the cross-sectional area of the dust particle, *i.e.* where *P* is the perimeter of the dust particle. However, the aspect ratio is related to the square of the longest projection length of the dust particle over the cross-sectional area of the dust, *i.e.* where *A* is the cross-sectional area and *L*_proj_ is the longest projection length of the dust particle. The shape factor resembles the major-to-minor axes ratio of the ellipsoid that is the best fit to the particle. The aspect ratio and the shape factor could not be correlated analytically in terms of functional form. The data corresponding to the geometric features of the dust particles reveal that the dust particles have arbitrary shapes and sizes. However, the average size of the dust particle (1.2 μm) gives rise to a shape factor in the order of 1.55. The ratio becomes almost three for the large-sized dust particles (≥10 μm). Table 1 provides EDS data (wt%) for the dust particles, while Fig. 7 shows an X-ray diffractogram of the dust particles. The dust particles contain various elements and compounds. The elemental composition of the small-sized dust particles changes slightly; in this case, oxygen and chlorine contents attain slightly larger values than those of the larger particles. X-ray diffractogram peaks for iron coincide with the aluminium and silicon peaks and the sodium and potassium peaks are likely to form due to sea salt, since the dust particles are obtained in the region close to the Gulf Sea. The sulfur content in the peak could be associated with calcium in the form of anhydrite or gypsum (CaSO_4_); however, the iron peak is likely to be related to clay-aggregated hematite (Fe_2_O_3_). Moreover, the dust particle adhesion on the hydrophobic surface is assessed using tangential force measurement using the AFM probe. In this case, the tangential force represents the force required to remove the dust particle from its position on the hydrophobic surface. In reality, the dust particles may roll off the inclined hydrophobic surface under gravitational potential.

**Fig. 6:** SEM micrographs of dust particles: (a) various sizes of dust particles, and (b) small-sized dust particles attach at large particle surfaces and form clusters.

**Table 1:** Elemental composition of dust (wt%) determined by energy dispersive spectroscopy (EDS)

	Si	Ca	Na	S	Mg	K	Fe	Cl	O
Size ≥ 1.2 μm	12.4	8.4	2.3	1.2	2.5	0.8	1.1	0.6	Balance
Size < 1.2 μm	10.2	7.3	2.8	2.2	1.4	1.5	1.1	1.3	Balance
Dust residues	12.5	6.1	1.1	0.8	1.2	0.5	0.3	0.2	Balance

**Fig. 7:** X-ray diffraction pattern of dust particles.

Consequently, the adhesion of the dust particles becomes necessary to ensure the dust particles deposited on the surface remain after the hydrophobic surface is inclined. The AFM cantilever tip faces a strain (in the friction mode) due to an obstacle along its path and the cantilever arm (tip) undergoes deflection. The slope of the deflection of the tip is demonstrated to be proportional to the force applied onto the cantilever arm of the AFM probe. This relation can be expressed as *F* = *kσ*Δ*V*,^36^ where *k* represents the spring constant of the cantilever tip (N m^−1^), *σ* corresponds to the slope of the displacement over the recorded probe voltage (Δ*z*/Δ*V*, m V^−1^), and Δ*V* is associated with the voltage recorded during the scanning of the AFM tip in the contact mode. The calibration of the probe reveals that *kσ* = 1.29375 × 10^−7^ nN mV^−1^. Consequently, the AFM cantilever data in friction mode shown in Fig. 8 result in an adhesion force in the order of 0.2 × 10^−5^ nN for dust size of about 1.0 μm. The weight of such a dust particle is in the order of 0.253 × 10^−5^ nN. Consequently the inclination of the hydrophobic surface by 5° gives rise to a gravitational force along the surface direction in the order of 0.02205 × 10^−5^ nN, which is considerably smaller than the adhesion force obtained from AFM probe data. Therefore, the dust particles remain on the inclined hydrophobic surface. However, when the inclination angle of the hydrophobic surface exceeds 55°, the dust particles roll off the surface.

**Fig. 8:** Atomic force microscope probe response for dust removal from the functionalized silica particle deposited surface; an atomic force microscope image of the dust particles is also shown.

Nevertheless, in the experiment, the inclination angle of the surface is considered to be 5°; hence the dust particle attaches on the surface.

### Droplet motion on inclined hydrophobic surface

Droplet dynamics on a hydrophobic surface are governed mainly by the contact angle and contact angle hysteresis. The contact angle hysteresis (*θ*_R_ − *θ*_A_, where *θ*_R_ is the droplet receding angle and *θ*_A_ is the droplet advancing angle) adversely contributes to the droplet movement, *i.e.* it increases the droplet pinning on the surface. On the other hand, the inclination of the hydrophobic surface generates a gravitational force while causing the droplet to roll and slide on the surface. In the case of a droplet in motion, the drag force due to pressure and friction influences and retards the motion while lowering the droplet acceleration on the inclined surface. Moreover, the shear force formed between the inclined surface and the flow in the droplet fluid, due to the droplet fluid being under gravitational potential, also adversely contributes to the droplet acceleration. On the other hand, as the forces balance among the gravitational and retention forces due to droplet pinning, drag, and shear under the rate of fluid strain at the droplet interface between the droplet fluid and the surface, if an imbalance favours the inertial gravitational potential, the droplet rolls off and/or slides on the inclined surface. However, the droplet motion is affected by the droplet bulging/wobbling (puddling) on the surface.^37^ The size of the droplet becomes important for rolling because of the puddle thickness, which is related to the droplet diameter. In this case, for a droplet diameter smaller than the capillary length ( where *κ*^−1^ represents the capillarity length, *σ* corresponds to the surface tension of the droplet fluid, *ρ* is the fluid density, and *g* represents the gravitational acceleration), the droplet rolls like a spherical marble without going through large puddling. However, the centre of mass of the droplet changes during the rolling as the droplet puddles. In addition, the droplet contact angle hysteresis, due to variation in the advancing and receding angles, changes because of droplet puddling. Therefore, the retention force on the hydrophobic surface changes during the puddling of large-sized droplets. The puddle thickness was introduced and formulated previously;^38,39^ in which case, the puddle thickness is  where *θ* corresponds to the droplet contact angle. A large-sized droplet under rolling motion suffers from elastic deformation on the inclined hydrophobic surface and the inertial force resulting from the force balance along the surface defines the droplet acceleration during rolling. The formulation of droplet acceleration based on force balance was presented in the earlier study,^28^ but the resulting equations are provided briefly for completeness of the argument. After consideration, the force balance equation for a rolling droplet on an inclined surface can be expressed as:^28^1where *m* represents the droplet mass; *δ* is the inclination angle of the hydrophobic surface; *F*_ad_, *F*_τ_, and *F*_f_ are the retention, shear, and frictional force between the surface and the droplet during rolling, respectively; *D*_a_ is the air drag force; *R* is the droplet radius; and *ω* is the angle of rotation. The equation for the retention force is:^28,29^2where *γ*_LV_ represents the surface tension of the liquid on the solid surface, *f* is the solid fraction (solid–liquid contact fraction due to surface texture), *D* is the droplet diameter prior to deformation (the same area as the ellipse), *θ*_R_ is the receding angle, and *θ*_A_ is the advancing angle. The frictional force due to the shear stress developed between the droplet liquid and the hydrophobic surface can be expressed as:4where *A*_w_ is the droplet contact area (*A*_w_ = π*r*^2^, where *r* is the contact area radius of the droplet), *μ* is the droplet fluid viscosity, *V*_d_ is the flow velocity in the droplet fluid, and *y* is the distance normal to the contact surface. As the droplet behaves like a solid rotating marble, the frictional force between the droplet and the hydrophobic surface can be written using the friction coefficient and the normal force, *i.e.*:

5 *F*_f_ = *μfF*_n_

where *μ*_f_ is the friction coefficient of the hydrophobic surface and *F*_n_ is the normal force, which is of the same order as the weight of the droplet (mg). The friction coefficient of the hydrophobic surface is obtained through the measurement of the AFM probe deflection data and the friction coefficient is found to be about 0.03. The drag force related to the flow resistance during the droplet rolling on the inclined hydrophobic surface can be formulated after assuming an equivalent spherical body to the droplet. In this case, the drag force (*D*_a_) can be written as *D*_a_ ≅ 1/2*C*_d_*ρ*_a_*A*_c_*U*_T_^2^, where *C*_d_ corresponds to the drag coefficient^40^ and *U*_T_ represents the air velocity opposing the droplet. It can be assumed that the air flow velocity is of the same order as the droplet translation velocity on the hydrophobic surface; hence, *U*_T_ ≅ *V*, where *V* represents the droplet translational velocity. Combining the influencing forces in the force balance equation (eqn (1)), the rotational speed of the droplet on the inclined surface becomes:6

Fig. 9 shows the rotational speed of the droplet predicted from eqn (6) and obtained from the high-speed camera data for various droplet volumes and a 5° inclination angle of the hydrophobic surface. It is evident that both results are in agreement and small differences between the results are related to experimental errors, which are in the order of 4%, and the assumptions made in the formulation, such as a spherical body in the drag force calculations and avoiding the sliding effect of the droplet on the surface during droplet rolling. Nevertheless, the difference between the results is small. The experiments are repeated twelve times to ensure the repeatability of the acceleration data. In addition, the trend of the rotational speed agrees with that obtained from the earlier work.^28^

**Fig. 9:** Rotational speed predicted from analytical relation and obtained from high-speed camera data on an inclined hydrophobic surface for a 40 μL water droplet. Inclination angle of surface is 5°.

The droplet kinetic energy under rotational motion should also satisfy the energy balance along the inclined surface. In this case, droplet puddling gives rise to work done, due to the geometric change induced by the Laplace pressure variation inside the droplet, which needs to account for the dissipative work during the droplet rolling. Consequently, droplet puddling, particularly for large-volume droplets, gives rise to potential energy dissipation during droplet rolling. In addition, the frictional losses because of droplet pinning and air drag should be accommodated in the energy equation to account for the potential energy dissipation of the droplet. The governing equation for the energy balance yields:

7 Δ*E*_Tot_ − Δ*E*_Diss_ = Δ*E*_Kin_

where Δ*E*_Tot_ corresponds to the potential energy of the particle at any location on the inclined hydrophobic surface and Δ*E*_Tot_ = *mg*Δ*h* (*m* is the mass of the droplet, *g* is the gravitational acceleration, and Δ*h* is the elevation between the droplet location and the reference level). *E*_Diss_ is the energy dissipation because of friction, adhesion, shear and air drag forces acting on the droplet during its movement on the hydrophobic surface. The energy dissipated (*E*_Diss_) is of the same order as Δ*E*_friction_ + Δ*E*_deformation_ + Δ*E*_retention_ + Δ*E*_shear_ + Δ*E*_air-drag_. Here, Δ*E*_friction_ is the energy dissipated due to shear between the droplet fluid and the hydrophobic surface, Δ*E*_deformation_ is the energy dissipation during puddling of the droplet (where the mass centre of the droplet changes), Δ*E*_retention_ is associated with the energy dissipation due to adhesion and friction during the droplet movement on the hydrophobic surface, and Δ*E*_air-drag_ is the energy dissipation due to the air drag generated during the droplet movement on the hydrophobic surface. The energy dissipation due to friction between the droplet and the surface can be written as Δ*E*_friction_ = *μ*Δ*LF*_n_, where *μ* is the dynamic friction coefficient between the water droplet and the hydrophobic surface, Δ*L* is the distance along the inclined hydrophobic surface, and *F*_n_ is the normal force due to the droplet weight. However, the energy dissipated due to droplet puddling (volumetric deformation) can be formulated using the droplet diameter in terms of the volumetric deformation; hence, it yields  where ∀p corresponds to the droplet volume, *γ*_L_ represents the droplet fluid surface tension and *D*_h_1__ and *D*_h_2__ are the hydraulic diameters of the droplet along the length scale Δ*L* on the surface due to puddling. The energy dissipated under the adhesion force can be described in terms of the droplet adhesion; hence, it yields:  where *θ*_A_ and *θ*_R_ are the dynamic advancing and receding angles of the droplet during its motion along the length scale Δ*L* on the inclined hydrophobic surface. The frictional loss in the droplet fluid due to the shear rate along the length scale Δ*L* on the hydrophobic surface can be formulated using the rate of fluid strain, which yields:  where *A*_w_ is the contact area (*A*_w_ = π*r*^2^, where *r* is the three-phase-contact radius), *μ*_t_ is the fluid dynamic viscosity, *V*_d_ is the velocity of flow in the droplet fluid, and *y* is the distance normal to the droplet liquid contact surface. Energy dissipated due to air drag can be formulated as:  where *K*_L_ represents the loss coefficient due to air drag. The tangential velocity (*U*_T_) is determined from the droplet angular speed (*ω*, eqn (6)) after incorporating the instant hydraulic radius of the droplet at any location on the hydrophobic surface, *i.e. D*_H_/2, which is the instant hydraulic diameter of the droplet. Therefore, the energy balance for the droplet yields:8

Eqn (8) can be used to predict the droplet translational velocity on the inclined hydrophobic surface. Fig. 10 depicts the droplet translational velocities predicted from eqn (8) and obtained from the high-speed camera data along the hydrophobic surface for different droplet volumes. The predictions of the droplet velocity and the measured data are in good agreement. However, as the distance along the hydrophobic surface increases, the difference between the predicted droplet translational velocity and the experimental data becomes slightly large. The differences between the results are associated with the assumptions made during the analytical formulation of the translational velocity and experimental errors. Nevertheless, both results are in good agreement. In the early period of droplet movement, due to the rapid acceleration of the droplet under gravitational influence, the translation velocity increases sharply. As the distance along the hydrophobic surface increases, the droplet velocity attains an almost steady value. The attainment of the steady droplet translational velocity is attributed to the energy balance between the energy dissipation and kinetic energy change, which becomes almost steady along the hydrophobic surface. In this case, increasing droplet acceleration increases the frictional drag and the shear rate at the interface between the droplet fluid and the solid surface. In addition, the dissipation work, due to droplet puddling, attains an almost steady value with increasing distance along the hydrophobic surface. It should be noted that the work dissipated (due to puddling) reduces because of the difference between the droplet maximum and minimum heights during the droplet movement along the hydrophobic surface. This can be seen from Fig. 11, in which the maximum droplet height variation along the hydrophobic surface is shown for three different droplet volumes. Increasing the droplet volume increases the droplet height oscillation in the early period of droplet movement. As the droplet moves along the inclined hydrophobic surface, the maximum height difference reduces, which is true for all droplet volumes considered. The gravitational force acting on the droplet volume works in favour of droplet puddling; however, the surface tension force reduces the puddle size. Consequently, the balance between the gravitational force and the surface tension force influences the droplet puddle thickness. During the droplet puddling on the hydrophobic surface, the centre of the droplet mass is lowered by a distance *λ* from the hydrophobic surface. The difference of the potential energy between the spherical and puddled droplets can be approximated as *σ*^2^ ≅ *ρgR*^3^, where *R* is the droplet radius and *γ*_f_ is the surface tension of the droplet liquid.^41^ The three-phase contact length on the surface due to droplet puddling can be related to: The minimization of the potential energy difference due to spherical and puddled droplets of the same radius in terms of the three-phase contact length yields: *ρgR*^3^*λ* ∼ *γ*_f_*l*^4^/*R*^2^. Hence, the three-phase contact length for the puddled droplet takes the form:  which is similar to that reported in the earlier study.^41^ Here,  corresponds to the capillary length. Incorporating the mathematical arrangements in the potential energy minimization formulation (*ρgR*^3^*λ* ∼ *γ*_f_*l*^4^/*R*^2^), the shift in the length scale occurring in the centre of mass of the droplet (*λ*) becomes:  The puddling of the droplet alters the maximum height, as seen from Fig. 11; *i.e.* the droplet height variation (the difference in the maximum and the minimum droplet heights within one complete droplet rolling cycle) is in the order of 0.40 mm. This agrees with the value obtained from the relation  which is of the order of 0.48 mm for a 3.1 mm diameter droplet. In addition, the displacement of the droplet mass centre (*λ*) increases with the droplet radius (*R*); hence, droplet wobbling increases with increasing droplet volume. The dynamic receding angle increases slightly as the droplet moves along the hydrophobic surface, which is more pronounced for large-volume droplets. This situation can be seen in Fig. 12, in which the advancing and receding angles with distance are shown for three droplet volumes. This, in turn, increases the pinning force slightly while altering the droplet puddling along the surface. In addition, the droplet wobbling and large change in the droplet height in early droplet motion on the hydrophobic surface result in energy dissipation while adversely influencing the increase in droplet kinetic energy.

**Fig. 10:** Translational velocity of droplets on a 5° inclined hydrophobic surface obtained from high-speed camera data.

**Fig. 11:** Maximum and minimum tip height variation of droplets in clean and dusty surfaces during wobbling on a 5° inclined hydrophobic surface.

**Fig. 12:** Water droplet hysteresis (difference between advancing and receding angles) along a 5° inclined hydrophobic surface for various droplet volumes.

Consequently, as the distance increases along the hydrophobic surface, the increase in the droplet velocity becomes gradual, which can be observed from Fig. 11. As the droplet height reduces along the hydrophobic surface, dissipation of energy becomes less due to work done because of the change in the volumetric centre of the droplet. Hence, the droplet kinetic energy continuously increases along the surface despite this increase becoming gradual. On the other hand, the rotational speed of the droplet increases sharply upon droplet formation on the hydrophobic surface and as the distance increases the rotational speed increase becomes gradual. This situation can be seen from Fig. 9, in which the rotational speed predicted from eqn (6) and that obtained from the high-speed camera data are shown. The rotational Bond number ( where *ρ* is the water density, *R* is the droplet radius, *ω* is the angle of rotation and *σ* is the surface tension) is associated with the square of the rotational speed; consequently, increasing the rotational speed enhances the rotational bond number. Since the rotational bond number represents the centripetal force over the surface tension force, increasing the centripetal force, due to the increase in rotational speed, stabilizes the volume centre of the droplet, *i.e.* the droplet wobbling reduces with an increase in the rotational bond number, consistent with the earlier study.^28^ Moreover, the velocity ratio due to tangential velocity over the translational velocity of the droplet (*ωR*/*V*) affects droplet wobbling because of its influence on the dynamic pressure change between the droplet interior and the surrounding atmosphere.^42^ The dynamic pressure change influences droplet wobbling for the condition  where Δ*ρ* represents the density difference between the droplet liquid and surrounding ambient air and *ρ*_a_ corresponds to the density of the ambient air surrounding the droplet. In the present study, *φ* varies between 800 and 950 depending on the droplet volume considered; hence, the influence of the dynamic pressure change does not significantly influence droplet wobbling, which is consistent with previous findings.^42^ The retention force due to droplet adhesion, friction, and air drag contributes to the drop slipping on the hydrophobic surface during droplet motion. Fig. 13 shows the slip velocity with the droplet position on the hydrophobic surface for different droplet volumes. The slip velocity is obtained from the difference between the translational and tangential rotational velocities of the droplet (=*V* − *ωr*_d_, where *r*_d_ is the instant droplet hydraulic radius at any location on the hydrophobic surface). The slip velocity remains almost the same for all locations of the droplet on the hydrophobic surface. However, the slip velocity increases slightly with increasing distance (position) on the hydrophobic surface. This behaviour is attributed to the increasing rotational speed with increasing distance; in this case, a slight increase in the receding angle of the droplet along the hydrophobic surface (Fig. 12), which reduces the translational velocity more than the tangential velocity of the droplet due to the rotation. Hence an increasing centripetal force, because of the increase in the rotational speed, not only reduces droplet wobbling, but also lowers the sliding velocity of the droplet on the hydrophobic surface.

**Fig. 13:** Slip velocity of droplets along a 5° inclined hydrophobic surface for various droplet volumes.

### Influence of dust particles on droplet motion on a hydrophobic surface

Fig. 14 depicts the droplet translational velocity along the hydrophobic surface in the presence of dust particles for three droplet volumes. In addition, the velocity data for a clean surface is also provided for comparison. The data presented in Fig. 14 are obtained from the high-speed camera during the experiments. The droplet translation velocity is reduced for the case of the dust particle deposited hydrophobic surface. This can be attributed to the friction and adhesion of the droplet on the hydrophobic surface. In this case, the dust particles act like obstacles on the droplet path while creating frictional resistance on the surface. In addition, the presence of the dust particles on the hydrophobic surface modifies the surface texture and alters the wetting state of the surface slightly; hence, the receding and advancing angles of the droplet during its motion on the surface can be modified. This, in turn, enhances the pinning force, due to droplet adhesion, on the surface. As the droplet moves along the surface, it picks up the dust particles from the surface and the droplet mass increases. Consequently, the gravitational potential increases with increasing droplet mass while influencing the droplet translational velocity on the surface. As the droplet size increases, the amount of dust particles picked up by the droplet increases, because of the large diameter of the three-phase contact line on the surface, and the droplet mass increases. This, in turn, enhances the influence of the gravitational potential and increases the droplet velocity. Therefore, the difference between the translational velocity due to a clean and a dust particle deposited surface becomes small for large-volume droplets, as can be seen from Fig. 14 after comparison of the translational velocity on the clean and dust particle deposited surfaces for different droplet volumes. Moreover, the droplet inertial force over the gravitational force is presented in terms of the Froude number.

**Fig. 14:** Droplet translational velocity on a dusty hydrophobic surface. Inclination angle of surface is 5°.

Fig. 15 depicts the Froude number (*V* is the velocity, *g* is the gravitational acceleration, and *L* is the distance) for different droplet volumes and the Froude number corresponding to the clean surface is also provided for comparison. The Froude number attains lower values for the droplet on the dusty hydrophobic surface than on the clean surface. This behaviour is attributed to the droplet translational velocity, which remains low for the hydrophobic surface with the presence of dust particles. In general, the Froude number attains low values as the droplet volume reduces.

**Fig. 15:** Froude number for droplets along a 5° inclined hydrophobic surface with the presence and absence of dust particles.

This is related to the droplet inertial force generated during the droplet motion on the hydrophobic surface; *i.e.* the velocity and the mass of the droplet reduce with reducing droplet size while lowering the droplet inertial force. Although the weight of the droplet adversely influences the Froude number, the Froude number increases with the droplet size because of the increase in the droplet inertial force. Hence, the influence of the droplet acceleration remains more critical than the gravitational acceleration on the dynamics of a droplet located on the hydrophobic surface. The droplet inertial force reduces for the dusty hydrophobic surface because of the low translational velocity of the droplet, which is more pronounced for a large-volume droplet. The droplet inertial force over the droplet surface tension force is also compared through the Weber number ( where *ρ* is the fluid density, *L* is the distance, *V* is the velocity, and *γ* is the air-liquid surface tension). Fig. 16 shows the variation in Weber number along the dust particle deposited hydrophobic surface for different droplet volumes. It should be noted that the variation in Weber number for the clean hydrophobic surface is also provided for comparison. The Weber number attains values within the order of unity when the translation velocity attains an almost steady increase.

**Fig. 16:** Weber number for droplets along a 5° inclined hydrophobic surface with the presence and absence of dust particles.

However, in the early departure of the droplet on the hydrophobic surface, where the distance along the hydrophobic distance is small, the inertial force remains less than the surface tension force. This is true for all the droplet volumes considered. As the translational velocity increases, the inertial force increases and the ratio of the inertial force over the surface tension force becomes greater than unity, which is more pronounced for large-volume droplets. It should be noted that increasing the droplet volume increases both the three-phase contact line on the hydrophobic surface and the droplet mass; however, the increase in the inertial force due to droplet acceleration remains larger than that of the surface tension force. Moreover, the presence of the dust particles lowers the surface Weber number appreciably. This is because of the attainment of a low translational velocity of the droplet when the dust particles are present on the hydrophobic surface (Fig. 14). Hence, the retarding of the droplet by the dust particles lowers the droplet inertia force considerably. Nevertheless, the Weber number attains values much less than that of the critical value for rolling droplets, which is estimated as We ∼11;^43^*i.e.* the large-sized droplets can break into multiple small droplets when the Weber number exceeds 11.

Fig. 17a shows a 3-dimensional optical image of the droplet path on the dust particle deposited hydrophobic surface. Most of the dust particles are picked up by the water droplet within its path on the hydrophobic surface. The size of the region where the droplet picks up the dust particles remains large for the large-sized droplets. In addition, droplet wobbling on the surface results in an oscillatory appearance on the surface where the dust particles are deposited. The width of the region cleaned by the droplet depends on the size of the three-phase contact line on the hydrophobic surface; *i.e.* the variation of the width of the cleaned region along the droplet path remains large for the large-sized droplet. Close examination of the 3-dimensional images reveals that some residues of the dust particles are observed along the droplet path on the hydrophobic surface. In order to assess the characteristics of the dust residues, SEM and EDS analyses are carried out. Fig. 18 shows an SEM micrograph of the dust residues while Table 1 gives the EDS data for the dust residues. The dust residues on the hydrophobic surface consist mainly of small dust particles (≤2 μm) but a few large-sized dust particles (≥5 μm) are also observed. The EDS data reveal that the oxygen content in the dust particle residues remains higher than that of the picked-up dust particles (Table 1). The densities of the dust particles collected and dust particle residues are assessed and the findings reveal that the density of the dust particles collected is in the order of 2800 kg m^−3^ while the density of the dust particle residues is in the order of 1600 kg m^−3^. Consequently, the dust particle residues are lighter in weight than the collected dust particles. In order to assess the water droplet cloaking on the dust particles, the study is further extended to include the behaviour of low surface energy dust particles when subjected to a rolling water droplet on the hydrophobic surface. The dust particles are functionalized by trichloro(1*H*,1*H*,2*H*,2*H*-perfluorooctyl) (PFOTS) through the vapour deposition technique, as described in the previous study.^44^ The functionalized dust particles are deposited onto the hydrophobic surface and droplet rolling experiments are repeated to observe the residues of the functionalized dust particles on the droplet path. Fig. 17b shows a 3-dimensional optical image of the functionalized dust particle residues on the hydrophobic surface along the droplet path. The functionalized dust particles are not all picked up by the water droplet and most of the dust particles remain on the hydrophobic surface as the residues of the dust particles. In order to assess the importance of water cloaking on dust particle removal by rolling droplets from the hydrophobic surface, the water cloaking velocities of the functionalized and normal dust particles are measured. The high-speed camera is used to measure the cloaking velocity of water on the dust particles. Fig. 19 shows images of water cloaking and the velocity of water cloaking on the normal dust particles. In addition, an image of the functional dust particles floating on the water surface is also shown; *i.e.* water cloaking did not take place on the functionalized dust particles even when the functionalized dust particle was placed on the water surface. The cloaking velocity increases rapidly in the early period and then becomes gradual with progressing time. In general, cloaking (spreading liquid onto the solid surface) takes place in steps. In the first step, the force balance between the surface tension and the shear at the interface of the dust particle and water forms a monolayer of water on the surface of the dust particle. The second step involves spreading, which progresses on the dust particle surface in accordance with Joos' law.^45^ The spreading velocity (*V*_sp_) of the water is related to  where *μ*_o_ corresponds to the dynamic viscosity of water, *ρ*_o_ represents the water density, and *S*_ow(a)_ is the water spreading coefficient on the dust particle.^46^ However, the dissipation force related to water spreading onto the dust particle can be formulated *via* the Ohnesorge number  where *a* represents the characteristic size of a dust particle,^46^ which can be assumed to be equivalent to the corresponding hydraulic diameter of the dust particle.^47^

**Fig. 17:** 3-dimensional optical image of the droplet path when normal dust particles and functionalized dust particles were deposited on a 5° inclined hydrophobic surface: (a) normal dust particles, and (b) functionalized dust particles. The circle represents dust residues on the droplet path.

**Fig. 18:** SEM micrograph of dust residues on a 5° inclined hydrophobic surface: (a) small-sized dust particles, and (b) complex-shaped dust particles.

**Fig. 19:** Temporal variation in water cloaking velocity on dust particles. Images of water cloaking on dust particles are also provided.

In the present case, the average-sized dust particle is in the order of 1.2 μm and using the data for water, the Ohnesorge number becomes greater than 1 (Oh > 1), which implies that a large dissipation force occurs during water cloaking of the dust particle. In addition, the rate of cloaking is related to the cloaking time in the form of ∼*k*_m_*t*^1/4^, where *k*_m_ is the cloaking factor.^47^ The cloaking is only possible when *k*_m_*t*^1/4^ > 1. The cloaking velocity in the initial cloaking stage (measured using the high-speed camera) is in the order of 0.29 m s^−1^ and the corresponding time is 0.05 s (Fig. 19). In addition, the cloaking velocity is inversely proportional to the cloaking time; in which case, the cloaking velocity decreases sharply with cloaking time (Fig. 19) in the form of ∼*Ct*^−0.5^, where *C* corresponds to a constant, which could vary with the dust particle shape, and *t* represents the cloaking time. In order to assess the water droplet cloaking onto the dust particles prior to picking them up from the hydrophobic surface during rolling, the cloaking time and the duration of the droplet passing through the dusty region are compared. In this case, the time corresponding to the distance travelled by the droplet over the wetting length (*l* ≅ 0.002 m for a 40 μL liquid droplet) with an average droplet translational velocity of 0.16 m s^−1^ is of the order of 12.5 milliseconds. The cloaking time for the same length is of the order of 6.5 milliseconds. Consequently, the water droplet cloaks the dust particles during rolling on the hydrophobic surface. Hence, the dust particles which are picked up by the water droplet are cloaked and wetted by the droplet liquid prior to its rolling cycle on the hydrophobic surface. On the other hand, the functionalized dust particles only attach onto the surface of the rolling droplet rather than being cloaked and picked up by the droplet from the hydrophobic surface. This situation can be observed from Fig. 20 in which optical images of the water droplet with the normal picked-up dust particles (Fig. 20a) and functionalized dust particles attached onto the droplet surface (Fig. 20b) are shown. Consequently, one of the main mechanisms for picking up the dust particles by the rolling droplet on the hydrophobic surface is closely related to the water cloaking of the dust particles during droplet rolling.

**Fig. 20:** Optical images of water droplets after rolling over a dusty 5° inclined hydrophobic surface: (a) normal dust particles picked up by the droplet and mixed with droplet fluid, and (b) functionalized dust particles attached on the droplet surface without mixing with the droplet liquid.

To assess the variation in the droplet cleaning performance on the hydrophobic surface for the various droplet volumes, the area ratio (*η*) is introduced, which corresponds to the area cleaned by the droplet over the total area corresponding to the rectangular geometry limited by the droplet diameter and the distance covered by the droplet. The droplet diameter is considered to be same as when the droplet is perfectly spherical. The area ratio represents the total area cleaned of dust particles by the droplet during the droplet motion on the hydrophobic surface. The area ratio with droplet volume is shown in Fig. 21a. Since the droplet undergoes wobbling, the wetted length/area (three-phase contact length/area) of the droplet changes on the hydrophobic surface. This situation can be seen from Fig. 21b, in which the maximum and minimum widths wetted by the water droplet on the surface are shown. This in turn results in some sections of the droplet path remaining dusty; *i.e.* the dust particles located in between the maximum and the minimum wetted width are not picked up by the droplet during its motion on the hydrophobic surface. The ratio of the clean surface area changes slightly with droplet volume; in this case, increasing the droplet volume slightly improves the ratio of the cleaned area on the droplet surface. However, further experiments may be needed to identify the optimum droplet diameter resulting in the maximum ratio of the cleaned surface.

**Fig. 21:** Area ratio of cleaned surface and droplet normalized width along a dusty 5° inclined hydrophobic surface and normalized droplet width on a hydrophobic surface: (a) area ratio corresponding to the actual area of dust particles picked up by a water droplet on the hydrophobic surface over a rectangular area associated with the droplet path when the equivalent droplet diameter (a spherical droplet prior to puddling) is incorporated along the same transverse length on the hydrophobic surface, and (b) normalized three-phase contact width (length) along the hydrophobic surface. The three-phase contact width is normalized by dividing by the equivalent droplet diameter (spherical droplet prior to puddling).

## Conclusions

Droplet motion on an inclined hydrophobic surface is considered in relation to environmental dust removal from surfaces. A polycarbonate wafer surface is crystallized in an acetone bath and silicon nano-particles are deposited on the crystallized polycarbonate surface using the deep coating technique. The conclusions derived from the present study are listed below:

The solution crystallization of the polycarbonate results in a hydrophobic wetting state on the surface with a droplet contact angle of 130° ± 4° and contact angle hysteresis of 36°. The silicon nano-particle deposition further improves the droplet contact angle (158° ± 2°) and lowers the contact angle hysteresis (2° ± 1°) on the crystallized surface. The roughness of the resulting surface is in the order of 4.2 μm, which is due to the formation of globules and fibrils on the polycarbonate surface after the solution-crystallization process.

Dust particles are collected from the local region of Dammam in the Kingdom of Saudi Arabia. The dust particles collected are analysed using SEM, EDS and XRD. The dust particles consist of various elements including Ca, Si, K, Na, Ca, Mg, Fe, O, and Cl. As the dust particle sizes reduce below 0.8 μm, the weight percentage of the elemental composition changes; hence, the oxygen content increases in the dust particles while the density of the dust particles is lowered from 2800 kg m^−3^ to 1600 kg m^−3^. The dust particles have various shapes and sizes. The average size of the dust particles is in the order of 1.2 μm.

The droplet rolls and slides on the inclined hydrophobic surface. The transverse velocity of the droplet increases with increasing droplet volume. This is attributed to the force balance, which favours the gravitational influence as the droplet mass increases due to increasing size. Droplet rotational speed also behaves similarly to increasing droplet volume. The retention force associated with the droplet adhesion, due to surface tension, interfacial shear between the droplet fluid and the hydrophobic surface, and air drag, influence the droplet acceleration along the hydrophobic surface. Increasing the retention force enhances droplet wobbling on the hydrophobic surface. In addition, increasing the droplet volume increases the puddle thickness of the droplet due to wobbling.

The presence of dust particles on the hydrophobic surface lowers the droplet tangential and transverse velocities. The sliding velocity of the droplet remains considerably small, at almost 13% of the droplet transverse velocity and it varies slightly along the hydrophobic surface. The rolling droplet picks up dust particles from the hydrophobic surface. The main mechanism associated with picking up the dust particles is related to the droplet water cloaking of the dust particles, which is much faster than the resident time of the droplet on the hydrophobic surface across the wetting length. In the case of functionalized dust particles, which do not undergo water cloaking, they are not picked up by the rolling droplet, but rather the particles attach onto the droplet surface; *i.e.* these particles do not mix with the droplet fluid. The area cleaned *via* droplet particle removal increases with an increase in the droplet volume.

The present study gives an insight into droplet dynamics on an inclined hydrophobic surface in the presence of dust particles. It also provides useful information on the self-cleaning of surfaces by a rolling droplet.

## Conflicts of interest

There are no conflicts to declare.

## Supplementary Material
